# Bone necrosis around dental implants: A patient treated with oral bisphosphonates, drug holiday and no risk according to serum CTX

**DOI:** 10.4317/jced.50698

**Published:** 2012-02-01

**Authors:** A J. Flichy-Fernández, S. González-Lemonnier, J. Balaguer-Martínez, Diego Peñarrocha-Oltra, Maria A. Peñarrocha-Diago, Jose V. Bagán-Sebastián

**Affiliations:** 1 Master in Oral Surgery and Implantology. Collaborating Professor of the Master in Oral Surgery and Implantology. Valencia University Medical and Dental School; 2 Associate Professor of Oral Surgery. Professor of the Master in Oral Surgery and Implantology. Valencia University Medical and Dental School; 3 Resident of the Master in Oral Surgery and Implantology. Valencia University Medical and Dental School; 4 Chairman of Stomatology. Valencia University Medical and Dental School. Head of the Service of Stomatology, Valencia University General Hospital

## Abstract

Osteonecrosis of the jaw (ONJ) may appear following certain oral surgery procedures in patients treated with oral bisphosphonates (OB). Guidelines for the treatment of these patients were set out in the American Association of Oral and Maxillofacial Surgeons (AAOMS) Position Paper on Bisphosphonate-Related Osteonecrosis of The Jaws (Position Paper) and Approved by the Board of Trustees in September 2006. For the AAOMS the placement of implants in these patients is not contraindicated. In addition, the serum C-terminal telopeptide bone suppressor marker (CTX) test is available to determine the risk of ONJ. A case is presented of ONJ in a patient with 6 months of OB discontinuation (“drug holiday”) before dental implant placement (following the guidelines of the AAOMS) and with no risk of osteonecrosis according to the serum CTX value (340 pg/ml). The wound healed favorably with complete healing at 7 months. In this case, the serum CTX test must be questioned as to its predictive value of ONJ, and more reliable markers of this risk are needed.

** Key words:**Bisphosphonates, dental implants, bone necrosis, serum CTX.

## Introduction

Osteonecrosis of the jaw (ONJ) is defined as the appearance of exposed bone in the maxillofacial region persisting for more than 8 weeks in patients with current or previous treatment with a bisphosphonate and no history of radiation therapy to the jaws (American Association of Oral and Maxillofacial Surgeons (AOMS)) (1).

According to the recommendations of the American Association of Oral and Maxillofacial Surgeons (AAOMS) (1), patients treated with oral bisphosphonates (OB) can receive dental implants. Marx et al. (2) found 2 cases of ONJ after placement of dental implants in patients taking OB for more than 3 years, without specifying whether the bisphosphonates were removed before surgery. In contrast, a review by Grant et al. (3), of 468 dental implants placed in 115 patients treated with OB, found no evidence of ONJ, only 2 implants failed, and success rates were comparable to patients not taking OB. Marx et al. (2) recommend the serum C- terminal telopeptide (CTX) blood test on an empty stomach, to assess the bone turnover/renewal suppression caused by OB, and so evaluate the risk of ONJ in patients who have been administered bisphosphonates for longer than 3 years. Less than 100 pg/mL is considered high risk, 100 pg/ml to150 pg/mL as moderate risk, between 150 pg/mL and 299 pg/mL as minimal risk, and greater than 300 pg/mL as no risk. On the other hand, Bagán et al. (4), found no significant relationship between this test and the number of exposed bone areas or the size of necrotic areas.

A case is presented of a woman who developed ONJ after placement of dental implants. The surgery was minimally invasive, carried out in a single phase and without complications. The guidelines of the AAOMS were followed, removing the OB 6 months before surgery and applying the serum CTX test, obtaining no risk of ONJ (according to Marx et al. (2).

## Case Report

The patient, a 61-year-old woman, presented to the Oral Surgery and Implantology Center for implant placement in the jaw. The patient’s medical history was positive for osteoporosis and she had been taking oral alendronate (70 mg/weekly) for 6 years and 6 months. After consultation with her orthopaedic surgeon, the medication was removed 6 months before making the serum CTX test. The result was 340 pg/mL, a value that corresponds with “no risk of ONJ” according to Marx et al. (4) criteria. Dental implants at 4.5 (series 4 of 13mm) and at 4.7 (series 3 of 13mm) (Defcon® Avantblast, Impladent, Senmenat, Barcelona, Spain) were placed, following the guidelines of the AAOMS of 2007. Surgery was minimally invasive, proceeding without incident, in a single phase, and placing crestal healing abutments (Fig. 1). Postoperative prescriptions consisted of amoxicillin 500 mg and 125 mg of clavulanic acid, 1/8h, for 7 days. Two weeks later, the patients presented an asymptomatic bone exposure of 1mm x 3mm, in the lingual area of implant 4.5 (Fig. 1D). A periapical radiography revealed a radiolucency distal of 4.5 (Fig. 2A). After 6 weeks with no tissue healing (criterion established by the AAOMS in 2007) and no remission of the bone necrosis, and after dismissing other possible causes of the lesion, the patient was classified as stage 1 of ONJ (exposed and necrotic bone in asymptomatic patients without evidence of infection). The treatment indicated by the AAOMS in these patients was established: rinses (0.12%, 3 times/day) and gel (0.2% 3 times/day) of chlorhexidine. The importance of maintaining good oral hygiene was emphasized to the patient.

**Figure 1:** Implant surgery in 4.5 and 4.7.A) Surgery site; B) Implant placement; C) Suturing; D) Ulcerated lesion lingual of 4.5 at 2 weeks (arrow); E) Ulcerated lesion lingual of 4.5 at 6 weeks after surgery (arrow); F) Complete healing at 7 months (arrow).

**Figure 2:** Radiographic control. A) Radiolucent image distal of 4.5 at 2 weeks of surgery (arrow); B) Bone resorption distal of 4.5 at 7 months (arrow); C) Maintenance of bone level at 1 year of prosthetic restoration (arrow).

Healing improved with this treatment, decreasing the area of exposed bone (Fig. 1E), with neither infection nor pain at any time. Treatment was maintained resulting in complete uneventful healing of the surgical site at 7 months. Clinical (Fig. 1F) and radiographic examination showed bone resorption distal of 4.5 (Fig. 2B), disap-pearance of the radiolucent image suggestive of necrotic bone, and being bone resorption higher in this region (distal of the implant in 4.5) than in unaffected regions (mesial of the implant in 4.5; mesial and distal of the implant in 4.7). At 1 year, no clinical or radiographic changes were observed (Fig. 2C); peri-implant bone level was stable. The prosthesis over implants was placed 3 months after healing (Fig. 3).

**Figure 3:** Check up at 1 year of prosthetic restoration A) Occlusal view; B) Lateral view.

## Discussion

We believe this is the first reported case of bone necrosis caused by OB in a patient with drug removal before surgery (following the guidelines of the AAOMS) and with no-risk serum CTX values (according to Marx et al.) (2).

Madrid and Sanz (5), in a systematic review, do not document any ONJ in patients taking OB (between 1 and 4 years) and with dental implants. For these authors, implant placement may be considered a safe procedure in patients taking OB. In contrast, Wang et al. (6) did present a case report of bone necrosis in dental implants in a patient taking OB for more than 10 years. Medication was not removed before surgery, treating the ONJ with chlorhexidine rinses 0.12% and azithromycin 500mg/3days. In the present study, OB was removed 6 months before placement of dental implants; healing was asymptomatic and an antibiotic was prescribed.

Marx et al. (2007) (4) state that CTX values over 300pg/mL indicate “no risk” of ONJ. The patient in the present study had a CTX value of 340pg/mL and still developed an ONJ. A study by Kunchur et al. (7), assessed the efficacy of the serum CTX test in determining the risk of ONJ in 348 patients taking OB; for these authors, the serum CTX test was not predictive in determining the risk of bone necrosis.

Official statements by the AAOMS in 2007 and 2009 (1) recommend that patients cease using OB 3 months prior to and 3 months after oral surgery to minimize the risk of ONJ. According to Marx et al. (2), if patients discontinued the medication 6 months before making the analysis a significant improvement in CTX values is produced in all cases, decreasing the risk of ONJ. In the present study, treatment with BF ceased 6 months before the surgery and still developed ONJ, being this possible due to the half-life of the BF in bone.

Regarding treatment of ONJ, Marx et al. (2), state that if the patient has no pain, then only chlorhexidine rinses 0.12% should be used until complete healing of the ONJ. If the patient is in pain, then antibiotic therapy is necessary, penicillin or levofloxacin, metronidazole, doxycycline, and erythromycin in cases of allergy to penicillin. In this case report, amoxicillin/clavulanic 3 times/day/7days was prescribed after surgery to avoid a possible complication. When the ONJ appeared the patient had no pain, so chlorhexidine rinses 0.12% were prescribed until complete healing, according to the criteria of Marx et al. (2).

Ruggiero et al. (8) state that radiographic changes do not become evident until significant bone involvement is produced. Periapical radiographs may not reveal significant changes in early stages of osteonecrosis. When extensive bone involvement is present, regions of mottled bone similar to that of diffuse osteomyelitis are noted (8). In this case report the initial periapical radiograph showed a radiolucent image of bone resorption, distal of 4.5 at 2 weeks, remaining at 12 months.

The surgery was minimally invasive, carried out in a single phase. There is no information in the literature on how to place implants in patients treated with OB; and this report raises the question as to whether surgery should be carried out in 2 phases, leaving the bone submerged, in these patients.

We believe this is the only case so far reported in the literature on a patient with bone necrosis in the jaw after dental implant placement, with minimally invasive, single phase surgery, removing oral bisphosphonates 6 months before the procedure (following AAOMS guidelines), and with a no risk value in the serum CTX test (according to Marx et al (2). This clinical case suggests that further studies are needed to support the capacity of the serum CTX test to predict the risk of ONJ.
